# Suppression of Neuroinflammatory and Apoptotic Signaling Cascade by Curcumin Alone and in Combination with Piperine in Rat Model of Olfactory Bulbectomy Induced Depression

This article has been retracted.

**DOI:** 10.1371/journal.pone.0061052

**Published:** 2013-04-17

**Authors:** Puneet Rinwa, Anil Kumar, Sukant Garg

**Affiliations:** 1 Pharmacology Division, University Institute of Pharmaceutical Sciences, UGC Centre of Advanced Study, Panjab University, Chandigarh, India; 2 Department of Pathology, Dr. Harvansh Singh Judge Institute of Dental Sciences and Hospital, Panjab University, Chandigarh, India; Universidade de São Paulo, Brazil

## Abstract

**Objectives:**

Bilateral destruction of the olfactory bulbs is known to cause behavioral changes analogous to symptoms of depression. Curcumin, a traditional Indian spice is currently being investigated in different psychiatric problems including depression. Dietary phytochemicals are currently used as an adjuvant therapy to accelerate their therapeutic efficacy. Therefore, the present study is an attempt to elucidate the neuroprotective mechanism of curcumin and its co-administration with piperine against olfactory bulbectomy induced depression in rats.

**Methods:**

Rats undergone olfactory bulbs ablations were analyzed after post-surgical rehabilitation period of 2 weeks. Animals were then treated with different doses of curcumin (100, 200 and 400 mg/kg; p.o.), piperine (20 mg/kg; p.o.) and their combination daily for another 2 weeks. Imipramine (10 mg/kg; i.p.) served as a standard control. Various behavioral tests like forced swim test (FST), open field behaviour and sucrose preference test (SPT) were performed, followed by estimation of biochemical, mitochondrial, molecular and histopathological parameters in rat brain.

**Results:**

Ablation of olfactory bulbs caused depression-like symptoms as evidenced by increased immobility time in FST, hyperactivity in open field arena, and anhedonic like response in SPT along with alterations in mitochondrial enzyme complexes, increased serum corticosterone levels and oxidative damage. These deficits were integrated with increased inflammatory cytokines (TNF-α) and apoptotic factor (caspase-3) levels along with a marked reduction in neurogenesis factor (BDNF) in the brain of olfactory bulbectomized (OBX) rats. Curcumin treatment significantly and dose-dependently restored all these behavioral, biochemical, mitochondrial, molecular and histopathological alterations associated with OBX induced depression. Further, co-administration of piperine with curcumin significantly potentiated their neuroprotective effects as compared to their effects alone.

**Conclusions:**

The present study highlights that curcumin along with piperine exhibits neuroprotection against olfactory bulbectomy induced depression possibly by modulating oxidative-nitrosative stress induced neuroinflammation and apoptosis.

## Introduction

Depression is one of the severe psychiatric disorders and has been estimated as the second biggest contributor of the global load of neurological diseases and disability for the year 2020 [1]. It is characterized by low mood, loss of interest in daily activities and marked reduction in pleasure activities. Although satisfactory progress has been made in understanding the pathophysiology of the disease but still there is need of a more valid animal model that mimics the manifestations of clinical depression and related problems.

Olfactory bulbectomy (OBX) has been widely used as an experimental model of depression [2]. Bilateral destruction of the olfactory bulbs caused complex alterations in behavioral, biochemical and cellular cascades, many of which are comparable to those seen in patients with major depression [2]. Bulb ablation results in anhedonia like state in sucrose preference test [3], increased hyperactivity in a novel environment [4] and increased immobility time [2]. Furthermore, OBX has also been reported to alter neurogenesis in several regions of brain, which is one of the putative pathogenic mechanisms to explain depression [5]. Studies have proved that damage to the hippocampal neurons can be reversed by chronic antidepressant treatments [6]. Since OBX-induced depressive symptoms respond to chronic, but not acute antidepressant treatment, thus OBX is considered as one of the best available models to evaluate antidepressant activity [2]. Interestingly, these OBX induced changes are independent of anosmia [7]. Since the olfactory bulb projects into different regions of the brain (cortex, amygdala and hippocampus), thus ablation of these bulbs results in neurodegeneration in the projection areas [2], which possibly explains OBX-induced behavioral changes. Although a lot of work is being carried out in this field, yet the therapeutic responses of newer antidepressant drugs are still not fully understood and hence often produce undesirable side effects. The approach towards development of safe and powerful antidepressant agents from traditional herbs may be a good novel therapeutic strategy for the treatment of depression.

Dietary and medicinal phyto-antioxidants these days are used as combination therapy with each other in order to limit their side effects and to increase their effectiveness. Curcumin, a polyphenolic compound derived from dietary spice turmeric, possesses diverse pharmacological effects including antioxidant [8], anti-inflammatory [9], and neuroprotective activities [10]. Curcumin have previously been reported to possess antidepressant-like effects in different experimental models [11], [12]. Studies have shown that antioxidant activities of curcumin are comparable to those of vitamin C and E [13]. Manganese complexes of curcumin are proved to have great capacity to protect brain lipids against peroxidation [14]. Studies from our laboratory also suggest that curcumin restored mitochondrial dysfunction and various mitochondrial enzyme complex activities [15]. Studies have documented a significant attenuated effect of curcumin on pro-inflammatory cytokines (TNF-a) [16]. Curcumin has also been known to enhance the level of brain derived neurotrophic factor (BDNF) [17]. Earlier, curcumin is also reported to significantly reduce stress induced increase in serum corticosterone levels in rats [18].

Piperine is a major alkaloidal constituent of black pepper. It is a powerful inhibitor of hepatic and intestinal glucuronidation, and increases the bioavailability of many drugs including curcumin [19], [20]. Since curcumin has a poor absorption rate and undergoes rapid metabolism which severely curtail its bioavailability, thus piperine has been tried as drug strategy with curcumin in the present investigation.

Based on this background, the present study has been designed with the aim to elucidate the neuroprotective mechanism of curcumin and its interaction with piperine against OBX induced behavioral, biochemical, mitochondrial, molecular and histopathological alterations.

## Materials and Methods

### Ethics Statement

The experimental protocols were approved by the Institutional Animal Ethical Committee (IAEC) of Panjab University (IAEC/282/UIPS/39 dated 30/8/12) and conducted according to the Committee for the Purpose of Control and Supervision of Experiments on Animals (CPCSEA) guidelines of Government of India on the use and care of experimental animals.

### Experimental Animals

Adult male Wistar rats (200–240 g) procured from Central Animal House, Panjab University, Chandigarh were used. Male rats were chosen to avoid the influence of female estrogen hormone on depression-like behavior. Animals were housed under standard (25±2°C, 60–70% humidity) laboratory conditions, maintained on a 12 hour natural day–night cycle, with free access to food and water. Animals were acclimatized to laboratory conditions before the experimental tests.

### Surgical Procedure (Olfactory Bulb Ablation)

Bilateral olfactory bulb ablation was performed as modified method described by different investigators [21]. Briefly, animals were anaesthetized with ketamine (75 mg/kg, i.p) and xylazine (5 mg/kg i.p) combination. All the surgical equipments were sterilized before use. The animals were fixed in a stereotactic frame (Stoelting Co., USA) and skull was exposed by a midline incision and burr holes (2 mm in diameter) were drilled 8 mm anterior to bregma and 2 mm on either side of the midline at a point corresponding to the posterior margin of the orbit of the eye. Both olfactory bulbs were removed by suction and holes were then filled with haemostatic sponge (AbGel, Absorbable gelatin sponge USP, Srikrishna Laboratories, India) and then scalp was stitched with absorbable sutures (Ethicon 4–0, Absorbable surgical sutures USP (Catgut), Johnson and Johnson, India). Sham-operated rats were treated in the same way, including piercing of the duramater but their bulbs were left intact. To prevent post surgical infection, the animals were received Sulprim injection^R^ (each ml containing 200 and 40 mg of sulphadiazine and trimethoprim respectively), intramuscularly (0.2 ml/300 g) once a day for 3 days of post-surgery. The OBX/Sham animals were housed singly in cages. The animals were then housed for two weeks (14 days) and given extra care to avoid aggressive behaviour, which might have developed otherwise. Drug treatments were started after a 14 days surgical rehabilitation period. Pictogram of the entire protocol is represented in Table 1.

**Table 1:** Experimental protocol design for olfactory bulbectomy experimental model.

Surgery and treatment schedule				Behavioral tests		
0^th^ day	0^th^–1^st^ day	2^nd^–14^th^ day	15^th^–28^th^ day	29^th^ day	30^th^ day	31^st^ day
Surgery	Recovery from surgery (Continuous care)	Rehabilitation period (Daily observation and handling)	Drug/vehicle treatment	Sucrose preference test	Open field exploration test	Forced swim test

### Drugs and Treatment Schedule

Curcumin and imipramine were purchased from Sigma Chemicals (St. Louis, MO, USA). Piperine was purchased from CDH, India. ELISA kit for TNF-α and caspase-3 were purchased from R&D Systems, USA, while Chemikine™ Brain Derived Neurotrophic Factor (BDNF) kit was procured from Millipore (USA). All other chemicals used for biochemical and mitochondrial estimations were of analytical grade. The animals were randomly divided into nine experimental groups with twelve animals in each. Entire study was conducted in multiple phases. First and second group was named as sham and OBX (ablation of olfactory bulbs) control group respectively. Curcumin (100, 200 and 400 mg/kg, p.o.) were treated as group 3–5 respectively. Piperine (20 mg/kg; p.o.) served as group 6. Co-administration of curcumin (100 and 200 mg/kg; p.o.) with piperine (20 mg/kg; p.o.) was categorized as group 7 and 8 respectively. Imipramine (10 mg/kg; i.p.) served as group 9. Curcumin and piperine were prepared in peanut oil and imipramine was dissolved in distilled water. Drugs were administered orally on the basis of body weight (5 ml/kg) and drug solutions were made freshly at the beginning of each day of the study protocol. Drugs were then administered once daily for a period of two weeks.

### Behavioral Assessments

#### Sucrose preference test

Rats were tested for sucrose consumption as described earlier [22]. Animals were housed individually throughout the test duration and presented two bottles simultaneously in the home cage, one containing a 1% w/v sucrose solution, and other containing standard drinking water during the 48 h training session. To prevent the preference to position, the location of the two bottles was varied during this period. After an 18 h period of food and water deprivation, an 8 h test session was conducted. The amount of liquid remaining in each bottle was measured at the end of the testing period. The sucrose preference score was expressed as percent of total liquid intake. Sucrose preference (SP) was calculated according to the following equation:.Where, SI = sucrose intake in grams and WI = water intake in grams.

#### Open field exploration

Open field behavior of rats was recorded in a circular arena of diameter 80 cm, surrounded by a 30 cm high wooden wall [23]. The arena painted white, was divided in to 25 small sections. Each rat was carefully placed in the centre of circular arena and allowed to explore the open field for 5 min. During this period, the ambulatory activity, in terms of the number of sections crossed, and the frequency of rearing was recorded along with defecation and licking episodes and values expressed as counts per 5 min.

#### Immobility period

Forced swim test was performed as described [24]. One day prior to the test, a rat was placed for conditioning in a clear plastic tank (45 cm×35 cm×60 cm) containing 30 cm of water (24±0.5°C) for 15 min (pretest session). Twenty-four hours later (test session); the total immobility period within a 5-min session was recorded as immobility scores (in sec). A rat was judged to be immobile when its hind legs were no longer moving and the rat was hunched forward (a floating position). The immobility time was recorded manually by an observer who was blind to the drug treatment.

### Biochemical Estimations

Immediately after the last behavioral test, animals were randomized into different sets; one set was used for the biochemical assays (n = 5/group). For biochemical analysis, animals were sacrificed by decapitation. Whole brain of each animal was put on ice and weighed. A 10% (w/v) tissue homogenates were prepared in 0.1 M phosphate buffer (*p*H 7.4). The homogenates were centrifuged at 10,000×g for 15 min and aliquots of supernatants were separated and used for biochemical estimation.

#### Lipid peroxidation

The extent of lipid peroxidation was determined quantitatively by performing the method as described by Wills [25]. The amount of malondialdehyde (MDA) was measured by reaction with thiobarbituric acid at 532 nm using Perkin Elmer Lambda 20 spectrophotometer (Norwalk, CT, USA). The values were calculated using the molar extinction co-efficient of chromophore (1.56×10 M^−1^ cm^−1^).

#### Nitrite

The accumulation of nitrite in the supernatant, an indicator of the production of nitric oxide was determined by a colorimetric assay with Greiss reagent (0.1% N-(1-napththyl) ethylene diamine dihydrochloride, 1% sulphanilamide and 5% phosphoric acid) [26]. Equal volumes of the supernatant and the Greiss reagent were mixed and the mixture was incubated for 10 min at room temperature in the dark. The absorbance was measured at 540 nm using Perkin Elmer Lambda 20 spectrophotometer (Norwalk, CT, USA). The concentration of nitrite in the supernatant was determined from sodium nitrite standard curve.

#### Reduced glutathione

Reduced glutathione in the brain was estimated according to the method of Ellman et al. [27]. Homogenate (1 ml) was precipitated with 1.0 ml of 4% sulfosalicylic acid and the samples were immediately centrifuged at 1200×g for 15 min at 4°C. The assay mixture contained 0.1 ml of supernatant, 2.7 ml of phosphate buffer of *p*H 8.0 and 0.2 ml of 0.01 M dithiobisnitrobenzoic acid (DTNB). The yellow color developed was read immediately at 412 nm using Perkin Elmer lambda 20 spectrophotometer (Norwalk, CT, USA). The results were expressed as micromoles of reduced glutathione per milligram of protein.

#### Catalase

Catalase activity was determined by the method of Luck [28], wherein the breakdown of hydrogen peroxide (H_2_O_2_) is measured at 240 nm. Briefly, the assay mixture consisted of 3 ml of H_2_O_2_, phosphate buffer and 0.05 ml of supernatant of tissue homogenate (10%), and the change in absorbance was recorded at 240 nm using Perkin Elmer lambda 20 spectrophotometer (Norwalk, CT, USA). The results were expressed as micromoles of H_2_O_2_ decomposed per milligram of protein/min.

#### Protein

The protein content was estimated by biuret method [29] using bovine serum albumin as a standard.

### Mitochondrial Enzyme Complex Estimations

Second set of animals (n = 5/group) were used for mitochondrial enzyme complex activities as described by Berman and Hastings [30]. The whole brain was homogenized in isolated buffer. Homogenates were centrifuged at 13,000 g for 5 min at 4°C. Pellets were re-suspended in isolation buffer with ethylene glycol tetraacetic acid (EGTA) and spun again at 13,000 g at 4°C for 5 min. The resulting supernatants were transferred to new tubes and topped off with isolation buffer with EGTA and again spun at 13,000 g at 4°C for 10 min. Pellets containing pure mitochondria were re-suspended in isolation buffer without EGTA.

#### Complex-I (NADH dehydrogenase activity)

Complex-I was measured spectrophotometrically by method of King and Howard [31]. The method involves catalytic oxidation of NADH to NAD^+^ with subsequent reduction in cytochrome *c.* The reaction mixture contained 0.2 M glycyl glycine buffer *p*H 8.5, 6 mM NADH in 2 mM glycyl glycine buffer and 10.5 mM cytochrome *c.* The reaction was initiated by addition of requisite amount of solubilised mitochondrial sample and followed absorbance change at 550 nm for 2 min.

#### Complex-II (Succinate dehydrogenase activity)

Complex-II was measured spectrophotometrically according to King [32]. The method involves oxidation of succinate by an artificial electron acceptor, potassium ferricyanide. The reaction mixture contained 0.2 M phosphate buffer *p*H 7.8, 1% BSA, 0.6 M succinic acid, and 0.03 M potassium ferricyanide. The reaction was initiated by the addition of mitochondrial sample and absorbance change was followed at 420 nm for 2 min.

#### Complex-III (MTT activity)

The MTT assay is based on the reduction of (3-(4, 5-dimethylthiazol-2-yl)-2, 5-diphenyl-H-tetrazolium bromide (MTT) by hydrogenase activity in functionally intact mitochondria. The MTT reduction rate was used to assess the activity of the mitochondrial respiratory chain in isolated mitochondria by the method of Liu et al. [33]. Briefly, 100 µl mitochondrial samples were incubated with 10 µl MTT for 3 h at 37°C. The blue formazan crystals were solubilised with dimethylsulphoxide and measured by an ELISA reader at 580 nm filter.

#### Complex IV (cytochrome c oxidase)

Cytochrome oxidase activity was assayed in brain mitochondria according to the method of Sottocasa [34]. The assay mixture contained 0.3 mM reduced cytochrome C in 75 mM phosphate buffer. The reaction was started by the addition of solubilized mitochondrial sample and the changes in absorbance were recorded at 550 nm for 2 min.

### Serum Corticosterone Estimations

#### Preparation of serum

Blood was collected (1.0 ml) between 8.00–9.00 AM through retro orbital bleeding in the test tube and allowed to clot at room temperature. The tubes were then centrifuged at 2000 rpm for 10 min. The straw colored serum was separated and stored frozen at −20°C.

#### Corticosterone assessment

For extraction of corticoster*one* the method of Silber et al. [35] was modified as described. 0.1–0.2 ml of serum was treated with 0.2 ml of freshly prepared chloroform: methanol mixture (2∶1, v/v), followed by 3 ml of chloroform instead of dichloromethane used in the procedure of Silber and its group [35]. The step of treatment of petroleum ether was omitted. The samples were vortexed for 30 sec and centrifuged at 2000 rpm for 10 min. The chloroform layer was carefully removed with the help of syringe with a long 16 gauge needle attached to it and was transferred to a fresh tube. The chloroform extract was then treated with 0.1 N NaOH by vortexing rapidly and NaOH layer was rapidly removed. The sample was then treated with 3 ml of 30 N H_2_SO_4_ by vortexing vigorously. After phase separation, chloroform layer on top was removed using a syringe as described above and discarded. The tubes containing H_2_SO_4_ were kept in dark for 30–60 min and thereafter fluorescence measurements carried out in fluorescence spectrophotometer (make Hitachi, model F-2500) with excitation and emission wavelength set at 472 and 523.2 nm respectively. The standard curve depicting the fluorescence yield versus corticosterone concentration was used for result analysis.

### Molecular Estimations

#### BDNF and TNF-α ELISA

The quantifications of BDNF and TNF-α were done with the help and instructions provided by Chemikine and R&D Systems immunoassay kits respectively. All samples were assayed in duplicate and absorbance was read on an ELISA plate reader (iMark™ Microplate absorbance reader, BIO-RAD) and the concentration of each sample was calculated by plotting the absorbance values on standard curve with known concentrations generated by the assay.

#### Caspase-3 colorimetric assay

Caspase-3, also known as CPP-32 is an intracellular cysteine protease that exists as a pro-enzyme, becoming activated during the cascade of events associated with apoptosis. The tissue lysates/homogenates can then be tested for protease activity by the addition of a caspase specific peptide that is conjugated to the color reporter molecule p-nitroaniline (pNA). The cleavage of the peptide by the caspase releases the chromophore pNA, which can be quantitated spectrophotometrically at a wavelength of 405 nm. The level of caspase enzymatic activity in the cell lysate/homogenate is directly proportional to the color reaction. The enzymatic reaction for caspase activity was carried out using R&D systems caspase-3 colorimetric kit.

### Histopathology of Brain Tissue

#### Tissue sections preparation

Remaining animals were deeply anaesthetized and perfused transcardially via the ascending aorta with cold phosphate buffered saline (0.1 M, *p*H 7.4) followed by fixative solution containing 4% (w/v) paraformaldehyde in 0.1 M PBS solution (*p*H 7.4). The whole brain was dissected out and fixed overnight at 4°C in the same buffer containing 4% (w/v) paraformaldehyde. The brain was then washed with 0.1 M PBS (*p*H 7.4) for 1 h, dehydrated in alcohol, and then embedded in paraffin wax. Serial coronal sections (5 µm thickness) of whole brain were then obtained.

#### Hematoxylin and Eosin (H&E) staining

The paraffin sections of whole brain (thickness 5 µm) were dewaxed and rehydrated with alcohol for hematoxylin-eosin (H&E) staining. The neurons in CA1 region of hippocampus and frontal cortex were examined under electron microscopy and photomicrographs were prepared.

### Statistical Analysis

Data are expressed as mean ± S.E.M. The data was analyzed by One-way ANOVA followed by Tukey's test. p<0.05 was considered as statistically significant. All statistical procedures were carried out using sigma stat Graph Pad Prism (Graph Pad Software, version 5, San Diego, CA).

## Results

### Effects of Curcumin, Piperine and their Combination on Sucrose Preference Test

Removal of olfactory bulbs caused significant reduction in sucrose consumption as compared to sham group. Curcumin (200, 400 mg/kg) significantly and dose dependently attenuated the reduction in sucrose consumption as compared to control (OBX) rats. Further, co-administration of piperine (20 mg/kg) with curcumin (100, 200 mg/kg) significantly potentiated the sucrose consumption as compared to their effects alone. The efficacy of the combination was comparable to that of imipramine (10 mg/kg) [F (11, 131) = 37.48 (p<0.01)] (Fig. 1).

**Figure 1:** Effects of curcumin, piperine and their combination on sucrose preference test (SPT). Values are expressed as mean *±* SEM. For statistical significance, ^a^ *P*<0.05 as compared to sham group; ^b^ *P*<0.05 as compared to OBX control;^ c^ *P<*0.05 as compared to OBX+C1; ^d^ *P<*0.05 as compared to OBX+C2; ^e^ *P<*0.05 as compared to OBX+P (One-way ANOVA followed by Tukey’s test). OBX, Olfactory Bulbectomy; C1, curcumin (100 mg/kg); C2, curcumin (200 mg/kg); C3, curcumin (400 mg/kg); P, piperine (20 mg/kg); I, imipramine (10 mg/kg).

### Effects of Curcumin, Piperine and their Combination in Open Field Performance Task

OBX rats exhibited a characteristic hyperactivity in the open field as depicted by increase in ambulation, rearing, defecation (number of fecal pellets) and reduction in grooming/licking episodes which was significant as compared to sham group. Curcumin (200, 400 mg/kg) treatment significantly reduced ambulation, rearing, defecation and improved grooming/licking episodes as compared to OBX group. Further, co-administration of piperine (20 mg/kg) with curcumin (100, 200 mg/kg) potentiated their protective effects on open field performance task which were significant as compared to their effects alone. The efficacy of the combination was comparable to that of imipramine (10 mg/kg). However, piperine (20 mg/kg) alone did not produce any significant effect on ambulation [F(11, 131) = 123.54 (p<0.01)], rearing [F(11, 131) = 152.14 (p<0.05)], grooming [F(11, 131) = 52.24 (p<0.05)] and defecation [F(11, 131) = 73.22 (p<0.05)] parameters as compared to OBX control (Table 2).

**Table 2:** Effect of curcumin, piperine and their combination on open field performance task.

Treatment(mg/kg)	Ambulation	Rearing	Grooming/lickingepisodes	Number of fecal pellets
**Sham**	102.6±5.95	28.2±2.49	8.4±1.26	0.5±0.18
**OBX control**	173.5±7.50^a^	43.8±2.18^a^	1.8±0.37^a^	4.8±0.51^a^
**OBX+ C1**	162.8±3.26	38.4±1.56	2.6±0.56	4.1±0.20
**OBX+ C2**	139.2±3.96^b^	34.6±1.41^b^	4.8±0.45b,c	2.6±0.28b,c
**OBX+ C3**	115.4±3.56c,d	31.8±1.07b,c	6.8±0.21c,d	1.2±0.20c,d
**OBX+ P**	169.6±4.34	44.2±3.56	1.8±0.56	4.4±0.64
**OBX+ C1+P**	134.6±4.57c,e	35.4±3.24b,e	4.6±0.87c,e	2.3±0.14c,e
**OBX+ C2+P**	118.4±5.56d,e	31.1±3.13c,e	6.4±0.93d,e	1.0±0.42d,e
**OBX+I**	110.4±5.11^b^	29.6±0.93^b^	7.3±1.17^b^	0.8±0.22^b^

Values are expressed as mean ± SEM. For statistical significance,

a P<0.05 as compared to sham group;

b P<0.05 as compared to OBX control;

c P<0.05 as compared to OBX+C1;

d P<0.05 as compared to OBX+C2;

e P<0.05 as compared to OBX+P (One-way ANOVA followed by Tukey’s test). OBX, Olfactory Bulbectomy; C1, curcumin (100 mg/kg); C2, curcumin (200 mg/kg); C3, curcumin (400 mg/kg); P, piperine (20 mg/kg); I, imipramine (10 mg/kg).

### Effects of Curcumin, Piperine and their Co-administration on Immobility Period

There was a significantly increase in the immobility period of OBX group as compared to sham treatment. Curcumin (200, 400 mg/kg) treatment significantly shortened immobility time as compared to OBX control. Curcumin (100 mg/kg) did not produce any significant effect on immobility period as compared to OBX group. Further, co-administration of piperine (20 mg/kg) with curcumin (100, 200 mg/kg) potentiated their protective effects (shortened immobility period) which were significant as compared to their effects alone. In addition, the efficacy of the combination was comparable to that of imipramine (10 mg/kg) F(11, 131) = 50.04 (p<0.01)] (Fig. 2).

**Figure 2:** Effect of curcumin, piperine and their co-administration on immobility period. Values are expressed as mean *±* SEM. For statistical significance, ^a^ *P<*0.05 as compared to sham group; ^b^ *P<*0.05 as compared to OBX control;^ c^ *P<*0.05 as compared to OBX+C1; ^d^ *P<*0.05 as compared to OBX+C2; ^e^ *P<*0.05 as compared to OBX+P (One-way ANOVA followed by Tukey’s test). OBX, Olfactory Bulbectomy; C1, curcumin (100 mg/kg); C2, curcumin (200 mg/kg); C3, curcumin (400 mg/kg); P, piperine (20 mg/kg); I, imipramine (10 mg/kg).

Effect of curcumin, piperine and their co-administration on lipid peroxidation (MDA), reduced glutathione (GSH), nitrite concentration and catalase enzymes level.

Olfactory bulbs ablation caused significant oxidative damage as evidenced by rise in MDA and nitrite levels, depletion of reduced GSH and catalase levels as compared to sham group. Chronic treatment with curcumin (200, 400 mg/kg) significantly attenuated oxidative damage (reduced MDA, nitrite levels, restoration of reduced GSH and catalase levels) as compared to OBX control. Further, co-administration of curcumin (100, 200 mg/kg) with piperine (20 mg/kg) significantly potentiated their antioxidant like effect which was significant as compared to their effect alone. The efficacy of the combination was similar to that of imipramine (10 mg/kg). However, piperine (20 mg/kg) alone did not produce any significant effect on LPO [F(11, 54) = 62.35 (p<0.01)], GSH [F(11, 54) = 49.12 (p<0.05)], Nitrite [F(11, 54) = 82.30 (p<0.01)] and Catalase [F(11, 54) = 40.21 (p<0.05)] activity as compared to control (Table 3).

**Table 3:** Effect of curcumin, piperine and their co-administration on lipid peroxidation (MDA), reduced glutathione (GSH), nitrite concentration and catalase enzymes levels.

Treatment(mg/kg)	LPO (mol of MDA/mgpr)(% of sham)	GSH (µmol of GSH/mgpr)(% of sham)	Nitrite (µg/ml)(% of sham)	Catalase (µmol of H_2_O_2_ hydrolysed/min/mgpr)(% of sham)
**Sham**	0.161±0.009 (100)	0.086±0.005 (100)	312±16.54 (100)	0.703±0.030 (100)
**OBX control**	0.530±0.025^a^ (329.2)	0.023±0.003^a^ (26.7)	770.8±13.96^a^ (247.1)	0.211±0.024^a^ (30.0)
**OBX+ C1**	0.442±0.035 (274.5)	0.031±0.002 (36)	683.5±11.84 (199.8)	0.233±0.045 (35.9)
**OBX+ C2**	0.379±0.020b,c (235.4)	0.045±0.005^b^ (52.3)	532.6±9.23b,c (170.7)	0.363±0.060b,c (51.6)
**OBX+ C3**	0.263±0.018c,d (163.4)	0.064±0.015c,d (74.4)	428.8±10.47c,d (150.3)	0.498±0.030c,d (58.0)
**OBX+ P**	0.506±0.030 (314.3)	0.028±0.0055 (32.6)	712.8±12.45 (228.5)	0.224±0.024 (31.9)
**OBX+ C1+P**	0.365±0.015c,e (226.7)	0.044±0.0025c,e (51.2)	545.4±15.78c,e (174.8)	0.354±0.043c,e (50.4)
**OBX+ C2+P**	0.274±0.015d,e (170.2)	0.062±0.0045d,e (67.4)	422.5±13.12d,e (154.6)	0.486±0.063d,e (60.6)
**OBX+ I**	0.176±0.022^b^ (109.3)	0.079±0.0039^b^ (91.9)	373±8.62^b^ (119.6)	0.573±0.027^b^ (77.2)

Values are expressed as mean ± SEM. For statistical significance,

a P<0.05 as compared to sham group;

b P<0.05 as compared to OBX control;

c P<0.05 as compared to OBX+C1;

d P<0.05 as compared to OBX+C2;

e P<0.05 as compared to OBX+P (One-way ANOVA followed by Tukey’s test). OBX, Olfactory Bulbectomy; C1, curcumin (100 mg/kg); C2, curcumin (200 mg/kg); C3, curcumin (400 mg/kg); P, piperine (20 mg/kg); I, imipramine (10 mg/kg).

### Effects of Curcumin, Piperine and their Co-administration on Mitochondrial Enzyme Complex Activity

There was a significant alteration in mitochondrial enzyme complex (I, II) activities (Fig. 3) and decreased number of viable cells (complex III) and levels of cytochrome C oxidase enzyme (complex IV) (Fig. 4) in OBX rats as compared to the sham group. Curcumin (200, 400 mg/kg) treatment significantly restored mitochondrial enzyme complex I, II activities and improved number of viable cells and levels of cytochrome C oxidase enzyme as compared to OBX control. However, curcumin (100 mg/kg) did not produce any significant effect on mitochondrial enzyme complex activities. Further, co-administration of piperine (20 mg/kg) with curcumin (100, 200 mg/kg) significantly potentiated its protective effects which was also significant as compared to their effects alone. The efficacy of the combination was comparable to that of imipramine (10 mg/kg). In addition, piperine (20 mg/kg) alone did not produce any significant effect on mitochondrial enzyme complex I [F(11, 54) = 30.88 (p<0.01)], II [F(11, 54) = 42.32 (p<0.05)], III [F(11, 54) = 38.0 (p<0.05)] and IV [F(11, 54) = 17.4 (p<0.05)] activities as compared to control.

**Figure 3:** Effect of curcumin, piperine and their co-administration on mitochondrial enzyme complex I and II activities. Values are expressed as mean *±* SEM. For statistical significance, ^a^ *P<*0.05 as compared to sham group; ^b^ *P<*0.05 as compared to OBX control;^ c^ *P<*0.05 as compared to OBX+C1; ^d^ *P<*0.05 as compared to OBX+C2; ^e^ *P<*0.05 as compared to OBX+P (One-way ANOVA followed by Tukey’s test). OBX, Olfactory Bulbectomy; C1, curcumin (100 mg/kg); C2, curcumin (200 mg/kg); C3, curcumin (400 mg/kg); P, piperine (20 mg/kg); I, imipramine (10 mg/kg).

**Figure 4:** Effect of curcumin, piperine and their co-administration on mitochondrial enzyme complex III and IV activities. Values are expressed as mean *±* SEM. For statistical significance, ^a^ *P<*0.05 as compared to sham group; ^b^ *P<*0.05 as compared to OBX control;^ c^ *P<*0.05 as compared to OBX+C1; ^d^ *P<*0.05 as compared to OBX+C2; ^e^ *P<*0.05 as compared to OBX+P (One-way ANOVA followed by Tukey’s test). OBX, Olfactory Bulbectomy; C1, curcumin (100 mg/kg); C2, curcumin (200 mg/kg); C3, curcumin (400 mg/kg); P, piperine (20 mg/kg); I, imipramine (10 mg/kg).

### Effect of Curcumin, Piperine and their Co-administration on Serum Corticosterone (CORT) Levels

OBX group of animals showed significant increase in serum CORT levels as compared to sham group. However, chronic treatment with curcumin (200 and 400 mg/kg) significantly attenuated the serum CORT levels as compared to OBX control. In-addition, co-administration of piperine (20 mg/kg) with curcumin (100, 200 mg/kg) significantly attenuated serum CORT levels which was also significant as compared to their effects alone. The efficacy of the combination was comparable to that of imipramine (10 mg/kg) [F(11, 54) = 177.0 (p<0.01)] (Fig. 5).

**Figure 5:** Effect of curcumin, piperine and their co-administration on serum CORT levels. Values are expressed as mean *±* SEM. For statistical significance, ^a^ *P<*0.05 as compared to sham group; ^b^ *P<*0.05 as compared to OBX control;^ c^ *P<*0.05 as compared to OBX+C1; ^d^ *P<*0.05 as compared to OBX+C2; ^e^ *P<*0.05 as compared to OBX+P (One-way ANOVA followed by Tukey’s test). OBX, Olfactory Bulbectomy; C1, curcumin (100 mg/kg); C2, curcumin (200 mg/kg); C3, curcumin (400 mg/kg); P, piperine (20 mg/kg); I, imipramine (10 mg/kg).

### Effect of Curcumin, Piperine and their Co-administration on Brain Tissue Necrosis Factor (TNF-α) and Caspase 3 Level

OBX rats showed significant increase in TNF-α and caspase 3 levels as compared to sham group. Curcumin treatment (200 and 400 mg/kg) significantly attenuated the levels of TNF-α and caspase 3 as compared to OBX control. However, curcumin (100 mg/kg) did not produce any significant effect on TNF-α and caspase 3 levels as compared to OBX group. Further, co-administration of piperine (20 mg/kg) with curcumin (100, 200 mg/kg) potentiated its protective effect (lowered TNF-α and caspase 3 levels) which was significant as compared to their effects alone. Further, the efficacy of the combination was comparable to that of imipramine (10 mg/kg). In addition, piperine (20 mg/kg) alone did not produce any significant effect on TNF-α [F(11, 54) = 47.14 (p<0.05)] (Fig. 6) and caspase 3 levels [F(11, 54) = 38.93 (p<0.01)] (Fig. 7) as compared to control.

**Figure 6:** Effect of curcumin, piperine and their co-administration on TNF- α activity. Values are expressed as mean *±* SEM. For statistical significance, ^a^ *P<*0.05 as compared to sham group; ^b^ *P<*0.05 as compared to OBX control;^ c^ *P<*0.05 as compared to OBX+C1; ^d^ *P<*0.05 as compared to OBX+C2; ^e^ *P<*0.05 as compared to OBX+P (One-way ANOVA followed by Tukey’s test). OBX, Olfactory Bulbectomy; C1, curcumin (100 mg/kg); C2, curcumin (200 mg/kg); C3, curcumin (400 mg/kg); P, piperine (20 mg/kg); I, imipramine (10 mg/kg).

**Figure 7:** Effect of curcumin, piperine and their co-administration on caspase 3 activity. Values are expressed as mean *±* SEM. For statistical significance, ^a^ *P<*0.05 as compared to sham group; ^b^ *P<*0.05 as compared to OBX control;^ c^ *P<*0.05 as compared to OBX+C1; ^d^ *P<*0.05 as compared to OBX+C2; ^e^ *P<*0.05 as compared to OBX+P (One-way ANOVA followed by Tukey’s test). OBX, Olfactory Bulbectomy; C1, curcumin (100 mg/kg); C2, curcumin (200 mg/kg); C3, curcumin (400 mg/kg); P, piperine (20 mg/kg); I, imipramine (10 mg/kg).

### Effects of Curcumin, Piperine and their Combination on Brain Derived Neurotrophic Factor (BDNF)

There was a significant reduction in BDNF levels of OBX animals as compared to sham group. Curcumin (200 and 400 mg/kg) treatment significant restored BDNF level as compared to OBX control. However, curcumin (100 mg/kg) treatment did not produce any significant effect on BDNF levels as compared to OBX control. Besides, combination of piperine (20 mg/kg) with curcumin (100, 200 mg/kg) significantly potentiated the protective effect (elevated BDNF level) as compared to their effects alone. Further, the efficacy of the combination was comparable to that of imipramine (10 mg/kg) [F(11, 54) = 50.99 (p<0.01)] (Fig. 8).

**Figure 8:** Effect of curcumin, piperine and their co-administration on BDNF levels. Values are expressed as mean *±* SEM. For statistical significance, ^a^ *P<*0.05 as compared to sham group; ^b^ *P<*0.05 as compared to OBX control;^ c^ *P<*0.05 as compared to OBX+C1; ^d^ *P<*0.05 as compared to OBX+C2; ^e^ *P<*0.05 as compared to OBX+P (One-way ANOVA followed by Tukey’s test). OBX, Olfactory Bulbectomy; C1, curcumin (100 mg/kg); C2, curcumin (200 mg/kg); C3, curcumin (400 mg/kg); P, piperine (20 mg/kg); I, imipramine (10 mg/kg).

### Effects of curcumin, piperine and their combination on histopathological changes in cerebral cortex and hippocampal CA1 region

Brain histology of sham animals showed typical histopathological structures of neurons in the cerebral cortex and CA1 region of the hippocampus. Removal of bulbs significantly enhanced levels of neuroinflammatory cells along with their degeneration (apoptosis) resulting in decreased cell density in both cerebral cortex and hippocampal CA1 region as compared with the sham group. However, treatment with curcumin (200 mg/kg) and (400 mg/kg) (not shown) attenuated these histological abnormalities. Combination of piperine (20 mg/kg) with curcumin (200 mg/kg) further restored histological alterations of neuronal cells as compared to curcumin (200 mg/kg) alone (Fig. 9).

**Figure 9:** Representative photomicrographs of cerebral cortex (A) and hippocampal CA1 region (B) of rat brain sections. Sections were stained with Haematoxylin and Eosin. Black arrows indicate neuroinflammation along with apoptotic cells 1: sham control: neurons are intact 2: OBX control: mild-moderate infiltration of inflammatory cells with large number of apoptotic cells 3: treated with curcumin (200 mg/kg): slight inflammation of neurons with less apoptotic cells 4: treated with curcumin (200 mg/kg) +piperine (20 mg/kg): neurons are preserved. (HE stain×250).

## Discussion

Olfactory bulbectomy (OBX) is a well established and widely used experimental model for studying the pathogenetic-mechanism of depression [2]. Ablation of olfactory bulbs generate many biochemical and cellular alterations that are similar to clinically depressed patients [36] and can be restored by several pharmaco-therapeutic interventions [2].

In the present study, OBX rats exhibited a characteristic hyperactivity in the open field paradigm and increased immobility time in the forced swim test, predicting symptoms associated with model of depression. These behavioral findings are very much in conformity with the previous studies on OBX rats [2]. Further, chronic administration of curcumin significantly and dose dependently reduced the immobility time in OBX treated rats. Similarly, curcumin also attenuated the hyperactivity associated with open field in OBX rats. The protective effect of curcumin was comparable to that of imipramine, which served as a positive control in the experiment. These behavioral observations are in agreement with the previous work examining the effects of chronic antidepressant treatment in OBX rats [37]. OBX model may also mimic different psychiatric symptoms found in clinically depressed patients. One of such symptoms i.e., anhedonia (loss of interest or pleasure) is a characteristic feature of endogenous depression [3]. Sucrose preference is regarded as an indicator of anhedonia-like condition [38]. In the present investigation OBX rats showed significant reduction in sucrose preference when compared to sham group, indicating a state of anhedonia. Further, curcumin in a dose dependent manner significantly restored the decrease in sucrose preference; thereby showing its antidepressant-like effects. This result is consistent with the reports from previous studies [4]. All these behavioral tests respond selectively to chronic curcumin treatment thus mimicking the clinical time course of antidepressant action.

Chronic stress activates hypothalamic–pituitary–adrenal (HPA) axis [39] and increases the levels of blood corticosterone in rats [40], similar to the human cortisol [41]. In our study, chronic stress induced by removal of olfactory bulbs resulted in significant rise in the serum corticosterone levels indicating hyperactivity of the HPA-axis [42]. Since increase in the corticosterone levels may lead to the behavioral alterations including depression-like symptoms [43], therefore it is possible to suggest that OBX-induced behavioral alterations observed in present study may be due to the increased levels of the serum corticosterone. However, chronic treatment with curcumin restored the elevated levels of serum corticosterone in OBX rats. These results are in accordance with the previous finding which showed that chronic curcumin administration attenuates stress-associated increased serum corticosterone levels [18].

Oxidative stress is an emerging focus of research, and plays a crucial role in the pathogenesis of depression [44]. Ablation of olfactory bulbs is reported to be associated with production of oxygen reactive species and saturation of antioxidant enzymes [45]. A significant increase in lipid peroxidation and marked decrease in the activity of reduced glutathione and antioxidant enzymes in the brain of OBX rats were found [45]. Studies on patients suffering from depression have shown decreased lipid peroxidation and antioxidant enzymes levels which returned to normal after antidepressant treatment [46]. Similarly, in the present study OBX animals also showed a significant increase in lipid peroxidation and a marked decrease in the activity of reduced glutathione and catalase enzyme. Curcumin attenuated lipid peroxidation [47] and restored endogenous antioxidant profile [48] showing its powerful radical scavenging property [49]. In this study, OBX rats showed a significant increase in nitrite levels thereby implicating endogenous brain nitric oxide in the neurobiology of depression [50]. This is further confirmed from clinical reports of depressed patients showing an elevated plasma nitrate levels [51]. Further, curcumin significantly reduced nitrosative stress by inhibiting elevated nitrite levels in brains of OBX rats. Curcumin has also been reported to inhibit *i*NOS expression [49] and particularly scavenge NO-based radicals [52], thereby signifying its potential against increased nitrite levels. The beneficial effects of curcumin against both oxidative and nitrosative stress are in accordance with the previous findings from our laboratory [53].

Mitochondrial oxidative damage is based on the fact that mitochondrial respiratory chain is the major sources of superoxide anion (O_2_^+^) generation [54]. Energy production in mitochondria is catalysed by protein complexes, namely NADH-ubiquinol oxidoreductase (complex-I), succinate-ubiquinol oxidoreductase (complex-II), ubiquinol cytochrome c oxidoreductase (complex-III) and cytochrome C oxidase (complex IV) [54]. In the present study OBX caused impairment in different mitochondrial enzymes complex activities. These results are in accordance with the previous findings from our laboratory [15]. Besides, mitochondrial impairment may generate excess of nitric oxide (NO) which further leads to oxidative damage [55]. Moreover, evidence suggests that mitochondria progressively gets damaged and loses their functional integrity due to reactive oxygen species (ROS) which thereby enhances oxidative damage [56]. This suggests that mitochondria dysfunction might be the key factor for the production of ROS which further leads to oxidative damage in OBX induced depression.

In addition to oxidative and nitrosative stress, OBX induced depression is also linked to the generation of inflammatory cytokines like TNF-α [57]. In our study we found elevated levels of TNF-α following OBX suggesting inflammatory reaction accompanied by neuronal damage [58]. This was later attenuated by chronic curcumin treatment in a dose-dependent manner which attributes to its potent anti-inflammatory properties [59]. Our findings are supported by observations from Cho et al. [16] who found a significant reduction of inflammatory cytokines (TNF-α) on treatment with curcumin. Apart from increased neuroinflammation, we also found significant enhancement in levels of apoptotic factor, caspase-3 in OBX animals, suggesting a role of apoptotic pathway in OBX-induced depression. Our findings are in concurrence with Hall and Macrides [60], who found neuronal cell death in different brain regions following olfactory bulbectomy. We found that treatment with curcumin significantly inhibited caspase-3 activity in OBX rats, which is further supported by studies from Bharti et al. [61]. These results are further evidenced through histopathological studies which show presence of a large number of inflammatory and apoptotic cells leading to mild-moderate neurodegeneration in OBX rats. Studies from Nesterova et al. [62] reported a significant degeneration in neurons of the temporal cortex and hippocampus following olfactory bulbectomy. Curcumin later showed marked improvement in the histopathology of neurons in both cortex and hippocampal neurons of OBX animals thereby displaying its neuroprotective effects.

The neurotrophin hypothesis of depression predicts that a downregulation of brain-derived neurotrophic factor (BDNF) is involved in the pathogenesis of depression [63]. Furthermore, studies from Koo et al. [5] have demonstrated a decreased brain neurogenesis in OBX animals. In the present investigation, OBX rats showed a significant decrease in BDNF levels, thereby showing a reduced neurogenesis, a putative pathogenic mechanism in depression. However, curcumin treatment stimulated neurogenesis and expression levels of the neurotrophic factors BDNF in OBX rats. These results are consistent with findings from other laboratories [64]. Thereby it can be suggested that behavioral alterations observed after OBX (decreased sucrose preference, hyperactivity in open field and increased immobility period) are due to neurodegeneration of various brain structures [65], [66].

Poor oral bioavailability of curcumin limits its therapeutic utility. Curcumin undergoes extensive reduction through alcohol dehydrogenase, followed by conjugations at various tissue sites mainly in liver and intestine [67]. Since piperine is a well known inhibitor of hepatic and intestinal glucuronidation therefore it is reported to increase the bioavailability of several drugs including curcumin [20]. In the present investigation, we witnessed a profound increase in neuroprotection effects of curcumin in combination with piperine, in olfactory bulbectomized animals indicating that piperine might have increased the bioavailability of curcumin. In addition to its inhibitory effect on hepatic and intestinal glucuronidation, piperine has also been reported to have many other actions viz; anti-depressant [68], anti-apoptotic [69], anti-inflammatory [70], anti-oxidative [71] and neuroprotectant [72]. However, in our study piperine per se did not produce any neuroprotective effect which might be due to difference in the dose, duration of treatment and pathologies of different experimental models involved in depression. Further, beneficial effects of piperine per se treatment against severe neurodegeneration and behavioral deficits associated with olfactory bulbectomy rat model have not been reported so far. To the best of our knowledge, this is also the first study which reports the inhibitory effect of piperine on hepatic and intestinal glucuronidation in olfactory bulbectomy rat model. In this study we unleashed the benefits of the combination by assessing significant changes in behavioral, biochemical, mitochondrial, molecular and histopathological parameters. The strength of this study lies in the fact that the combination of piperine and curcumin were strongly neuroprotective in assessment of different parameters of the study.

In conclusion, the findings of the present study raised the possibility that oxidative-nitrosative stress-mediated inflammatory cascade may have resulted in activation of apoptotic signaling pathways and contributed to the neurodegeneration associated with depression like symptoms in rat model of olfactory bulbectomy. Curcumin on the other hand showed anti-apoptotic, neuroprotective actions due to its multiple effects viz strong anti-inflammatory, radical scavenging and neuromodulating properties. Piperine on the other hand proved to be a potent bioavailability enhancer and to a greater extent has resolved the problems of intestinal degradation related to curcumin. However, further studies are required to fully understand the curcumin’s action in neurodegenerative process associated with depression and to establish its clinical effectiveness in patients suffering from depression and related disorders. Together, co-administration of curcumin and piperine may provide a useful natural adjuvant in the antidepressant therapy.
